The article "Multivariate Analysis and Prediction Model Construction for Dermatoscope Use by Chinese Dermatologists via an Online Survey" was published in 2024. Journal: Skin Res Technol.

# Multivariate Analysis and Prediction Model Construction for Dermatoscope Use by Chinese Dermatologists via an Online Survey

**DOI:** 10.1111/srt.70087

**Published:** 2024-10-09

**Authors:** Mengguo Liu, Feng Xu

**Affiliations:** ^1^ Department of Dermatology Huashan Hospital Fudan University Shanghai China

**Keywords:** Chinese dermatologists, dermatoscope, prediction model, questionnaire survey

## Abstract

**Background:**

The use of dermatoscopes is constantly increasing globally, but to date, there are no studies on the use of dermatoscopes by Chinese dermatologists.

**Objective:**

To determine factors influencing the use of dermatoscopes in China.

**Methods:**

A web‐based questionnaire was designed by the Department of Dermatology at Huashan Hospital affiliated with Fudan University and was published online via the Shanghai Wheat Color Intelligent Technology Company, China. In 2019 and 2022, 1581 and 1507 dermatologists, respectively, were recruited and completed the questionnaire online.

**Results:**

In China, the application rate of dermatoscopy is higher in eastern provinces than in western and remote areas. The proportion of doctors from public tertiary hospitals is the highest, with females being the majority. The age range of 30–40 years has the highest proportion, the proportion of doctors with professional titles of attending physician or above is the highest, and the proportion of doctors with a bachelor's degree or above is the highest.

**Conclusions:**

By improving the education and professional standards of doctors, providing more training opportunities, simplifying access, and promoting dermatoscopy in grassroots hospitals, we can increase the confidence of dermatologists in the use of dermatoscopy.

## 1 Introduction

Dermatoscopy is a globally recognized technique for assisting in the diagnosis of skin diseases and is more accurate and visible than the naked eye [1]. The advantages of dermatoscopy are its convenience and noninvasiveness. Dermatoscopy can provide more visual information about pathological changes within the skin, which requires specialized dermatoscopy training and professional knowledge for analysis [2].

Initially, dermatoscopy was most commonly used to assist in the diagnosis of melanoma and nonmelanoma skin tumors [3, 4, 5]. However, dermatoscopy has been used to diagnose various other types of skin diseases, including infectious skin diseases, inflammatory skin diseases, hair diseases, and nail diseases [6, 7, 8, 9]. In addition, dermatoscopy can monitor changes in lesions over time and monitor changes in skin lesions during drug treatment [10, 11].

The use of dermatoscopes is increasing globally, and many recognized guidelines have been established. Research data show that there are significant differences in the usage rates of dermatoscopes between European and American countries, ranging from 48% to 98.5% [12, 13, 14, 15]. However, there is currently no research on the use of dermatoscopes by Chinese dermatologists and their influencing factors. Therefore, the purpose of this study was to evaluate the knowledge of Chinese dermatologists about dermatoscopy through a web‐based questionnaire. In addition, we constructed a predictive model to screen out the most meaningful influencing factors.

The article "Multivariate Analysis and Prediction Model Construction for Dermatoscope Use by Chinese Dermatologists via an Online Survey" was published in 2024. Journal: Skin Res Technol.

## 2 Methods

### 2.1 Study Design

This study was initiated and sponsored by the Department of Dermatology at Huashan Hospital affiliated with Fudan University. We designed a web‐based questionnaire by reviewing the literature and consulting the Chinese Skin Image Database (CSID) expert committee. Technicians from Shanghai Wheat Color Intelligent Technology Company provided technological support. The skin imaging group of the Department of Dermatology at Huashan Hospital was responsible for conducting this survey.

### 2.2 Online Survey Platform

We published the questionnaire on the UMER Doctor platform for 2 weeks (from August 1 to 15, 2019; and from October 1 to 15, 2022). The UMER Doctor application is the largest online learning platform for dermatologists in China. Dermatologists from the UMER Doctor platform were recruited to complete the questionnaire online and were prompted to complete the questionnaire in 20 min. The participating dermatologists also provided their demographic information, professional title, and hospital name and level.

### 2.3 Division of Observations

In this questionnaire, we classified age groups according to the following guidelines: < 30 years old, 30−39.9 years old, 40−49.9 years old, and ≥ 50 years old. Hospitals in China are mainly divided into 3‐tier systems (primary, secondary, and tertiary hospitals) based on their ability to provide medical care, medical education and conduct medical research, along with additional services such as community health service stations, private clinics, and village clinics. The professional titles of dermatologists in China include chief physicians, associate chief physicians, attending physicians, resident physicians, and others. To measure the level of attention of dermatologists towards dermatoscopy, we designed the following questions: (1) Whether to use a dermatoscope: Yes or No. (2) Frequency of using dermatoscopes: always, often, sometimes, never. (3) Dermatoscope sources: personal purchase, hospital purchase, both personal and hospital purchase, and others. (4) Dermatoscope type: handheld contact type, handheld noncontact type, workstation, mixture. (5) Confidence level: confident, not confident. (6) The reasons for not using these tools are as follows: They are uninterested, difficult to obtain, useless, not trained, and time‐consuming.

The article "Multivariate Analysis and Prediction Model Construction for Dermatoscope Use by Chinese Dermatologists via an Online Survey" was published in 2024. Journal: Skin Res Technol.

### 2.4 Statistical Analysis

The data in this study are categorical variables expressed in terms of the number of cases (*n*) and composition ratio (%), and comparisons between different groups were conducted via the *χ* ^2^ test. We used the “glmnet” software package LASSO regression for variable selection, conducted multiple logistic regression to construct a predictive model, and drew subject working characteristic curves, calibration curves, and clinical decision curves to evaluate the performance of the predictive model. All statistics in this study were completed via R 4.3.2, a double‐sided test, and a test level of *α* = 0.05.

## 3 Results

### 3.1 Basic Data of the Participating Dermatologists

#### 3.1.1 Analysis of the Provinces in Which the Dermatologists Participated in the Survey

A total of 1581 dermatologists from 32 provinces/municipalities/autonomous regions participated in the questionnaire survey in 2019 (Figures 1 and 2). The top three participating provinces were Guangdong Province (139 persons), Shandong Province (117 persons), and Fujian Province (115 persons). The last three regions were the Macao Special Administrative Region and Xizang Autonomous Region (1 person), Qinghai Province (7 persons), and Hainan Province (9 persons). In 2022, 1507 dermatologists from 32 provinces/municipalities/autonomous regions participated in the questionnaire survey. The top three participating regions were Shandong Province (131 persons), Guangdong Province (107 persons), and Jiangsu Province (98 persons). The bottom three participating provinces were Guizhou and Hainan Provinces (8 persons), Qinghai Province (10 persons), and Gansu Province (17 persons).

**FIGURE 1:** Comparison of the number of participants in the survey between 2019 and 2022 in different provinces.

**FIGURE 2:** Basic characteristics of the respondents in 2019 and 2022.

#### 3.1.2 Age Analysis of the Dermatologists Who Participated in the Survey

In 2019, the average age of the dermatologists was 36.70 years (standard deviation of 8.08), with a median age of 36 years. In 2022, the average age of dermatologists was 35.37 years (standard deviation of 8.42), with a median age of 34 years.

#### 3.1.3 Gender Analysis of the Dermatologists Who Participated in the Survey

In 2019, the gender ratio of dermatologists was 631 males, accounting for 39.91%, and 950 females, accounting for 60.09%. In 2022, the male‐to‐female ratio of 1507 dermatologists was 406 males, accounting for 26.98%, and 1099 females, accounting for 73.02%.

The article "Multivariate Analysis and Prediction Model Construction for Dermatoscope Use by Chinese Dermatologists via an Online Survey" was published in 2024. Journal: Skin Res Technol.

#### 3.1.4 Analysis of the Educational Background of the Dermatologists Who Participated in the Survey

In 2019, there were 767 dermatologists with a bachelor's degree or below, accounting for 48.5%, and 815 with a master's degree or above, accounting for 51.5%. In 2022, there were 686 dermatologists with a bachelor's degree or below, accounting for 45.5%, and 821 with a master's degree or above, accounting for 54.5%.

#### 3.1.5 Analysis of the Professional Titles of the Dermatologists Who Participated in the Survey

In 2019, the titles of dermatologists included 447 resident physicians, accounting for 28.3%, 599 attending physicians, accounting for 37.9%, 318 deputy chief physicians, accounting for 20.1%, 116 chief physicians, accounting for 7.3%, 60 medical students, accounting for 3.8%, and 41 others, accounting for 2.6%. In 2022, the professional titles of dermatologists included 490 resident physicians, accounting for 32.5%, 574 attending physicians, accounting for 38.1%, 197 deputy chief physicians, accounting for 13.1%, 71 chief physicians, accounting for 4.7%, 103 medical students, accounting for 6.8%, and 72 others, accounting for 4.8%.

#### 3.1.6 Analysis of the Nature and Level of Hospitals Where Dermatologists Participated in the Survey

In 2019, the nature of the hospitals where dermatologists are located was as follows: 1450 physicians from public hospitals, accounting for 91.7%; 98 physicians from private hospitals, accounting for 6.2%; and 33 physicians from other hospitals, accounting for 2.1%. The level of the hospital is as follows: 1031 physicians from a tertiary hospital, accounting for 65.2%; 336 physicians from a secondary hospital, accounting for 21.3%; 58 physicians from a primary hospital, accounting for 3.7%; and 156 physicians from other hospitals, accounting for 9.9%. In 2022, the nature of the hospital where dermatologists are located is as follows: 1381 physicians from public hospitals, accounting for 91.6%; 110 physicians from private hospitals, accounting for 7.3%; and 16 persons from other hospitals, accounting for 1.1%. In terms of hospital level, 1042 physicians from third‐level hospitals, accounting for 69.2%, 296 physicians from second‐level hospitals, accounting for 19.6%, 39 physicians from first‐level hospitals, accounting for 2.6%, and 130 persons from other hospitals, accounting for 8.6%.

### 3.2 Analysis of the Use of Dermatoscopes by Dermatologists

#### 3.2.1 Analysis of the Use of Dermatoscopes by Dermatologists of Different Gender and Ages

In 2019, among the dermatologists who used dermatoscopes, 374 were males, accounting for 39.4%, and 575 were females, accounting for 60.5% (Table 1 and Figure 3). Age distribution: 30 years old: 205 physicians accounting for 21.6%, 30−39.9 years old: 451 physicians, accounting for 47.5%, 40−49.9 years old: 216 physicians, accounting for 22.7%, ≥ 50 years old: 77 physicians, accounting for 8.1%. In 2022, among the dermatologists who used dermatoscopes, 284 males accounted for 25.2%, and 843 females accounted for 74.7%. Age distribution: 30 years old: 374 physicians, accounting for 33.2%; 30−39.9 years old: 470 physicians, accounting for 41.7%; 40−49.9 years old: 216 physicians, accounting for 19.1%; ≥ 50 years old: 68 physicians, accounting for 6.0%.

The article "Multivariate Analysis and Prediction Model Construction for Dermatoscope Use by Chinese Dermatologists via an Online Survey" was published in 2024. Journal: Skin Res Technol.

**TABLE 1:** Comparison of dermatoscopy usage between 2019 and 2022.

	2019			2022		
	Use dermoscope *n* (%)	No use dermatoscope *n* (%)	*p*	Use dermoscope *n* (%)	No use dermatoscope *n* (%)	*p*
Gender			0.644			0.007
Male	374 (39.4)	256 (40.6)		284 (25.2)	122 (32.2)	
Female	575 (60.5)	375 (59.4)		843 (74.7)	256 (67.5)	
Age (years)			<0.001			<0.001
< 30	205 (21.6)	101 (16.0)		374 (33.2)	73 (19.3)	
30–39.9	451 (47.5)	268 (42.5)		470 (41.7)	155 (40.9)	
40–49.9	216 (22.7)	197 (31.2)		216 (19.1)	100 (26.4)	
≥ 50	77 (8.1)	62 (9.8)		68 (6.0)	51 (13.5)	
Education			0.011			<0.001
Undergraduate or below	485 (51.1)	281 (44.5)		428 (38.0)	243 (66.4)	
Master or above	465 (48.9)	350 (55.5)		698 (62.0)	123 (33.6)	
Hospital grade			0.088			<0.001
Third level hospital	600 (63.2)	431 (68.3)		871 (77.2)	171 (45.1)	
Secondary hospital	206 (21.7)	130 (20.6)		153 (13.6)	143 (37.7)	
First level hospital	37 (3.9)	21 (3.3)		19 (1.7)	20 (5.3)	
Other	106 (11.2)	49 (7.8)		85 (7.5)	45 (11.9)	
Professional title			0.079			<0.001
Resident physician	286 (30.1)	161 (25.5)		381 (33.8)	109 (28.8)	
Attending physician	348 (36.6)	250 (39.6)		417 (37.0)	157 (41.4)	
Deputy chief physician	192 (20.2)	126 (20.0)		136 (12.1)	61 (16.1)	
Chief physician	59 (6.2)	57 (9.0)		54 (4.8)	17 (4.5)	
Medical students	35 (3.7)	25 (4.0)		90 (8.0)	13 (3.4)	
Other	29 (3.1)	12 (1.9)		50 (4.4)	22 (5.8)	
Hospital nature			0.002			<0.001
Governmental hospital	890 (93.7)	560 (88.7)		1055 (93.5)	326 (86.0)	
Private hospital	44 (4.6)	54 (8.6)		65 (5.8)	45 (11.9)	
Other	16 (1.7)	17 (2.7)		8 (0.7)	8 (2.1)	
Whether training or not			0.853			<0.001
Yes	381 (40.1)	256 (40.6)		526 (46.6)	68 (17.9)	
No	569 (59.9)	375 (59.4)		602 (53.4)	311 (82.1)	
Whether confident or not			0.013			<0.001
Yes	251 (26.4)	203 (32.2)		434 (38.5)	24 (6.3)	
No	699 (73.6)	428 (67.8)		694 (61.5)	355 (93.7)	

**FIGURE 3:** Use of dermatoscopes by dermatologists in 2019 and 2022.

#### 3.2.2 Analysis of the Use of Dermatoscopes by Dermatologists With Different Educational Backgrounds and Professional Titles

In 2019, among the dermatologists who used dermatoscopes, 485 had a bachelor's degree or below, accounting for 51.1%, and 465 had a graduate degree or above, accounting for 48.9%. There are 286 resident physicians, accounting for 30.1%; 348 attending physicians, accounting for 36.6%; 192 deputy chief physicians, accounting for 20.2%; and 59 chief physicians, accounting for 6.2%. In 2022, there were 428 doctors with a bachelor's degree or below, accounting for 38.0%, and 698 doctors with a master's degree or above, accounting for 62.0%, who used dermatoscopes. There are 381 resident physicians, accounting for 33.8%, 417 attending physicians, accounting for 37.0%, 136 deputy chief physicians, accounting for 12.1%, and 54 chief physicians, accounting for 4.8%.

The article "Multivariate Analysis and Prediction Model Construction for Dermatoscope Use by Chinese Dermatologists via an Online Survey" was published in 2024. Journal: Skin Res Technol.

#### 3.2.3 Analysis of the Use of Dermatoscopes by Dermatologists From Hospitals of Different Natures and Levels

In 2019, 890 dermatologists used dermatoscopes in public hospitals, accounting for 93.7%, and 44 dermatologists in private hospitals, accounting for 4.6%. There are 600 physicians in tertiary hospitals, accounting for 63.2%, 206 physicians in secondary hospitals, accounting for 21.7%, and 37 physicians in primary hospitals, accounting for 3.9%. In 2022, there were 1055 dermatologists using dermatoscopes in public hospitals, accounting for 93.5%, and 65 dermatologists in private hospitals, accounting for 5.8%. There are 871 physicians in tertiary hospitals, accounting for 77.2%; 153 physicians in secondary hospitals, accounting for 13.6%; and 19 persons in primary hospitals, accounting for 1.7%.

#### 3.2.4 Analysis of the Frequency of Dermatologists Using Dermatoscopes

In 2019, among the dermatologists who participated in the survey, 950 (60.1%) used dermatoscopes, and 631 (39.9%) did not use them. Among them, 549 physicians (34.7%) frequently use it, 347 physicians (21.9%) sometimes use it, and 170 physicians (10.7%) rarely use it. In 2022, 1128 physicians (74.9%) used dermatoscopy, whereas 379 physicians (25.1%) did not use it. Among them, 732 physicians (48.6%) frequently use it, 340 physicians (22.6%) sometimes use it, and 164 physicians (10.9%) rarely use it.

#### 3.2.5 Analysis of the Sources and Types of Dermatoscopes Used by Dermatologists

In 2019, among the dermatologists who participated in the survey, 215 (13.6%) were purchased by individuals, 672 (42.5%) were purchased by hospitals, and 78 (4.9%) were purchased by both individuals and hospitals. A total of 465 (38.6%) were handheld contacts, 141 (11.7%) were handheld noncontacts, 538 (44.7%) were workstations, and 60 (5.0%) were hybrids. In 2022, 129 (8.6%) were purchased by individuals, 970 (64.4%) were purchased by hospitals, and 88 (5.8%) were purchased by both individuals and hospitals. A total of 573 (37.1%) are handheld contacts, 229 (14.8%) are handheld noncontacts, 669 (43.4%) are workstations, and 72 (4.7%) are hybrids.

The article "Multivariate Analysis and Prediction Model Construction for Dermatoscope Use by Chinese Dermatologists via an Online Survey" was published in 2024. Journal: Skin Res Technol.

#### 3.2.6 Analysis of the Confidence Level of Dermatologists in the Use of Dermatoscopy and the Reasons for Not Using Dermatoscopy

In 2019, 454 physicians (28.7%) were confident in using dermatoscopy, whereas 1128 physicians (71.3%) were not confident. In 2022, 458 physicians (30.9%) were confident in their use of dermatoscopy, whereas 1049 physicians (69.6%) were not confident.

In 2019, among the reasons for not using dermatoscopes, 9 physicians (0.9%) said they were not interested, 525 physicians (50.4%) said they were difficult to obtain, 19 physicians (1.8%) thought they were not helpful, 421 physicians (40.4%) thought they had not received any training, and 68 physicians (6.5%) believed it took too much time. In 2022, among the reasons for not using dermatoscopes, 33 physicians (3.7%) said they were not interested, 314 physicians (35.6%) said they were difficult to obtain, 57 physicians (6.5%) believed it was not helpful, 363 physicians (41.2%) believed they did not receive any training, and 114 physicians (12.9%) believed it took too much time.

### 3.3 LASSO Regression Screening Variables

This study included 10 possible influencing factors, including gender, age, education level, professional title, hospital level, hospital nature, investigation time, the confidence level in dermatoscopy technology when evaluating and judging characteristic structures under dermatoscopy, the confidence level in dermatoscopy technology when diagnosing skin lesions, and whether or not to receive dermatoscopy training, in the model for screening (Table 2). Each curve in Figure 4A represents the trajectory of changes in the coefficients of each candidate variable; as *λ* increases, the degree of model compression increases, and the number of candidate variables entering the model decreases. Figure 4B shows the process of 10× cross‐validation to determine the optimal *λ* value. The two dashed lines in the graph represent lambda‐min and lambda.1se. The dashed line on the left is lambda. min, which is the one selected in cross‐validation with the minimum cross‐validation error *λ* value. Lambda.1se is the addition of a standard error value based on lambda‐min. Usually, choosing the model corresponding to lambda.1se will be simpler and more interpretable. In this study, lambda.1se = 0.02162256 was chosen, and the variables included in the model were gender, age, education level, hospital level, survey time, the confidence level in dermatoscopy technology when evaluating and judging characteristic structures under dermatoscopy, the confidence level in dermatoscopy technology when diagnosing skin lesions, and whether patients received dermatoscopy training.

The article "Multivariate Analysis and Prediction Model Construction for Dermatoscope Use by Chinese Dermatologists via an Online Survey" was published in 2024. Journal: Skin Res Technol.

**TABLE 2:** LASSO regression screening variables.

		Not use dermatoscope (*N* = 1010)	Use dermoscope (*N* = 2078)	*p* value
Gender				<0.001
	Male	406 (40.2)	637 (30.7)	
	Female	604 (59.8)	1441 (69.3)	
Confidence in diagnosing characteristic skin lesion structures				<0.001
	Lack of confidence	650 (64.4)	190 (9.1)	
	Moderate confidence	247 (24.5)	1090 (52.5)	
	Confidence	113 (11.2)	798 (38.4)	
Confidence in diagnosing skin lesions				<0.001
	Lack of confidence	616 (61.0)	152 (7.3)	
	Moderate confidence	221 (21.9)	875 (42.1)	
	Confidence	173 (17.1)	1051 (50.6)	
Training				<0.001
	No	803 (79.5)	1054 (50.7)	
	Yes	207 (20.5)	1024 (49.3)	
Age				<0.001
	≤ 36 years	489 (48.4)	1304 (62.8)	
	> 36 years	521 (51.6)	774 (37.2)	
Education				<0.001
	Junior college	128 (12.7)	91 (4.4)	
	Bachelor degree	533 (52.8)	714 (34.4)	
	Master degree or above	349 (34.6)	1273 (61.3)	
Professional title				
	Chief physician	49 (4.9)	138 (6.6)	
	Deputy chief physician	194 (19.2)	321 (15.4)	
	Attending physician	427 (42.3)	746 (35.9)	
	Resident physician	277 (27.4)	660 (31.8)	
	Medical students	25 (2.5)	138 (6.6)	
	Other	38 (3.8)	75 (3.6)	
Hospital level				<0.001
	1 grade	57 (5.6)	40 (1.9)	
	2 B grade	64 (6.3)	53 (2.6)	
	2 A grade	274 (27.1)	241 (11.6)	
	3 B grade	120 (11.9)	183 (8.8)	
	3 A grade	363 (35.9)	1407 (67.7)	
Hospital nature				<0.001
	Governmental hospital	886 (87.7)	1945 (93.6)	
	Private hospital	99 (9.8)	109 (5.2)	
	Other	25 (2.5)	24 (1.2)	
Time				<0.001
	2019	631 (62.5)	950 (45.7)	
	2022	379 (37.5)	1128 (54.3)	

**FIGURE 4:** Construction of the prediction model for dermatoscope use by Chinese dermatologists. (A) Shrinkage coefficient plot. (B) Ten‐fold cross‐validation plot. (C) Prediction model ROC curve. (D) Prediction model calibration chart. (E) Clinical decision curve.

### 3.4 Logistic Regression Models

A total of 2078 of the 3088 dermatologists included in this study used dermatoscopes. The eight variables selected by LASSO regression were used as independent variables, and dermatoscopy was used as the dependent variable to establish a multivariate logistic regression model. The specific results are shown in Table 3. As shown in Figure 5, a column chart is drawn for visualization on the basis of the results of multiple factor logistic regression. Each predictor variable can project a score vertically onto the rating axis and then sum the scores of each predictor variable to obtain a total rating. The research object is the corresponding position found on the total rating axis, and the value projected vertically onto the risk axis is the probability of using dermatoscopy.

The article "Multivariate Analysis and Prediction Model Construction for Dermatoscope Use by Chinese Dermatologists via an Online Survey" was published in 2024. Journal: Skin Res Technol.

**TABLE 3:** Multivariate logistic regression analysis model.

Variable		OR(95% CI)	*p* value
Gender	Male	ref.	
	Female	0.84 (0.67, 1.05)	0.127
Age	≤ 36 years	ref.	
	> 36 years	0.79 (0.63, 0.98)	0.034
Confidence in diagnosing characteristic skin lesion structures	Lack of confidence	ref.	
	Moderate confidence	4.94 (3.52, 6.94)	< 0.001
	Confidence	6.37 (4.11, 9.86)	< 0.001
Confidence in diagnosing skin lesions	Lack of confidence	ref.	
	Moderate confidence	4.83 (3.40, 6.88)	< 0.001
	Confidence	4.68 (3.09, 7.07)	< 0.001
Training	No	ref.	
	Yes	2.31 (1.83, 2.91)	< 0.001
Education	Junior college	ref.	
	Bachelor degree	1.34 (0.92, 1.94)	0.122
	Master degree or above	2.09 (1.38, 3.14)	< 0.001
Hospital level	1 grade	ref.	
	2 B grade	1.59 (0.80, 3.17)	0.184
	2 A grade	1.54 (0.89, 2.67)	0.121
	3 B grade	2.26 (1.25, 4.08)	0.007
	3 A grade	5.06 (2.93, 8.75)	< 0.001
Time	2019	ref.	
	2022	2.31 (1.87, 2.85)	< 0.001

**FIGURE 5:** Nomogram of the probability of dermatologists using dermatoscopes.

### 3.5 Prediction Model Evaluation

The ROC curve is shown in Figure 4C, and the AUC and 95% CI of the prediction model were 0.89 (0.87−0.90). The optimal classification threshold for the model is 0.67, which means that the prediction probability is > 0.67 of the research subjects are classified as those who use dermatoscopes; otherwise, they are classified as those who do not use dermatoscopes. At this point, the corresponding sensitivity and specificity are 85.1% and 76.9%, respectively. The calibration chart is shown in Figure 4D. The dashed diagonal represents the ideal model, the solid line represents the actual performance of the model, and the closer the solid line is to the diagonal, the stronger the predictive ability of the model. The model exhibited good consistency and good predictive ability. The clinical decision curve results (Figure 4E) show that the model can benefit approximately 95% of the study subjects, indicating that at a higher probability threshold, the model provides a greater net benefit in deciding whether to use dermatoscopy and can provide greater decision support.

## 4 Discussion

In this study, from the perspective of geographical distribution, the use of dermatoscopes among the participants was more common in eastern coastal provinces, such as Guangdong, Shandong, Fujian, and Jiangsu, and less common in western and remote areas, such as Guizhou, Qinghai, Hainan, Gansu, and Xizang. There are regional differences in the use of dermatoscopes in China, and the use of dermatoscopes should be further promoted in western and remote provinces of China. From a gender perspective, in 2019 and 2022, female doctors accounted for a greater proportion of dermatoscopy use, which may be related to their preference for dermatology in their career choices. In terms of age, in 2019 and 2022, the median ages were 36 and 34 years, respectively. The proportion of doctors in the 30−40 years age group was the highest (47.5% and 41.7%, respectively), indicating that the majority of doctors using dermatoscopy were middle‐aged and young doctors. In terms of education and professional titles, in 2019 and 2022, the highest proportion of dermatoscopy users were those with a bachelor's degree or above, and those with attending physicians or above had the highest proportion. From the perspective of the nature and level of hospitals where doctors are located, the proportion of doctors in public and tertiary hospitals is the highest, whereas the proportion of doctors in private, secondary, and lower hospitals is relatively low. Therefore, it is necessary to further promote the use of dermatoscopes in grassroots hospitals and private hospitals.

The article "Multivariate Analysis and Prediction Model Construction for Dermatoscope Use by Chinese Dermatologists via an Online Survey" was published in 2024. Journal: Skin Res Technol.

We also found that in 2019 and 2022, 71.3% and 69.6% of dermatologists, respectively, lacked confidence in the use of dermatoscopes, with only 34.7% and 48.6% of doctors frequently using dermatoscopes in their diagnosis and treatment work. Among the reasons for not using dermatoscopes, in 2019 and 2022, they were mainly due to inability or difficulty in obtaining dermatoscopes (50.4% and 35.6%, respectively) and lack of training (40.4% and 41.2%, respectively).

In this study, we also used LASSO regression to screen eight variables (gender, age, education level, hospital level, survey time, the confidence level in dermatoscopy technology when evaluating and judging characteristic structures under dermatoscopy, the confidence level in dermatoscopy technology when diagnosing skin lesions, and whether to receive dermatoscopy training) as independent variables. Using dermatoscopy as the dependent variable, we established a multivariate logistic regression model. A simple, highly operational, and predictive model was constructed by constructing eight predictive factors and visualized through a nomogram to improve the convenience of clinical use. This is beneficial for increasing the usage rate of interventions by dermatologists, improving disease diagnosis accuracy and efficacy, and improving the patient experience. However, this study also has certain limitations, such as the inability to verify causality and the inability to conduct external data validation. Further data collection for external validation is needed in future research.

The article "Multivariate Analysis and Prediction Model Construction for Dermatoscope Use by Chinese Dermatologists via an Online Survey" was published in 2024. Journal: Skin Res Technol.

Socioeconomic factors significantly affect the availability and use of dermoscopy through multiple aspects, such as income level, medical security policies, educational resources, geographical location, social culture, economic development level, and industry trends. To promote the popularization and application of dermoscopy technology, it is necessary to fully consider the impact of these factors and take corresponding measures to improve the penetration rate and usage rate of dermoscopy. The following measures can be taken to improve the economics of dermoscopy equipment and reduce the cost of purchase and use; strengthen education and training to improve doctors' and patients' awareness and ability to use dermoscopy; adjust medical security policies to include dermoscopy examination in medical insurance coverage; and optimize the allocation of medical resources to ensure that all populations can access dermoscopy services fairly.

There is a positive correlation between the level of training in dermoscopy and confidence in the use of dermoscopy. Emphasizing this correlation can help advocate for more structured and systematic training programs, which not only help increase the popularity of dermatologists using dermoscopy but also significantly increase their diagnostic confidence in clinical practice. Such training programs should include in‐depth explanations of the basic principles of dermoscopy, guidance on practical operations, and regular evaluation and feedback to ensure that doctors can continuously improve their skills and diagnostic accuracy.

Different types of dermoscopy have different usage scenarios and preference differences in the hospital environment. Digital dermoscopy is more popular in large hospitals and specialized dermatology hospitals because of its high‐resolution image acquisition and storage capabilities, whereas handheld dermoscopy is more popular in primary care institutions because of its portability and affordability. The emergence of new dermoscopy technologies provides doctors with more choices and may further enhance diagnostic capabilities in different clinical environments. The development of customized dermoscopy technologies for different clinical environments in the future will help meet the practical needs of more doctors and promote the further development of dermatology technology.

Personal attitudes play a crucial role in the adoption of medical technology and the provision of medical services. For the adoption of new medical technology such as dermoscopy, personal attitudes not only affect patients' acceptance of the technology but also affect whether medical service providers are willing and able to effectively apply the technology. Therefore, to increase the adoption rate of dermoscopy, we need to focus on issues such as doctors' cognition, learning, and trust and actively address their psychological barriers and difficulties. By strengthening publicity and education, training support, policy guidance, and other measures, we can encourage medical service providers to actively adopt new technologies and improve the quality and efficiency of medical services.

The article "Multivariate Analysis and Prediction Model Construction for Dermatoscope Use by Chinese Dermatologists via an Online Survey" was published in 2024. Journal: Skin Res Technol.

The lack of longitudinal follow‐up in this study is an important limitation. Short‐term data collection may affect the predictive validity of the model, as short‐term data often provide information only at a certain point in time or within a short period of time and are not sufficient to fully reflect changes and trends over a longer period of time. Future research could consider conducting long‐term follow‐up surveys and collecting longitudinal data to gain a deeper understanding of the adoption process and long‐term effects of dermoscopy by health care providers.

This study captures data at only two time points, and there is a potential risk of overlooking potential time biases in the use of dermoscopy over time. First, recognizing the limitations of this study, we clearly noted this point in our discussion. Because the data were obtained at only two time points, they cannot fully reflect the long‐term trends or fluctuations in dermoscopy use. Second, despite only having two time points, through simple trend analysis, comparing the data at these two time points can provide a preliminary judgment that dermoscopy use has increased. Third, in the discussion section, we suggest that future studies increase the number of time points for data collection to assess the dynamic changes and long‐term trends in dermoscopy use more accurately. Finally, we carefully interpret the results. Owing to the risk of time bias, we emphasize the uncertainty of the research results, which may not fully reflect the actual situation.

This survey study was conducted before and after the COVID‐19 epidemic, and there were indeed some significant changes in the statistics of some variables between the two surveys. This change is closely related to many factors, such as changes in education and training models caused by the epidemic, changes in work pressure, and changes in the supply and accessibility of dermoscopy equipment. In addition, technological progress and increased marketing and publicity of dermoscopy equipment may have increased doctors' willingness and confidence in the use of dermoscopy. The update of dermoscopy training content and improvements in training participation have enabled doctors who have received training to apply dermoscopy more effectively for diagnosis, changing the overall statistics of dermoscopy use. Hospitals may have adjusted relevant policies, such as providing more support or incentives to doctors who use this new dermoscopy technology, thus promoting the popularization and use of dermoscopy.

The article "Multivariate Analysis and Prediction Model Construction for Dermatoscope Use by Chinese Dermatologists via an Online Survey" was published in 2024. Journal: Skin Res Technol.

## 5 Conclusion

Dermatoscopy has important application value in clinical practice because it improves diagnostic accuracy, reduces unnecessary biopsy or surgical resection, improves patient satisfaction, and promotes the effective use of medical resources. Therefore, we should further promote and apply dermatoscopy technology to provide patients with better medical services. By developing targeted dermoscopy education programs and starting by identifying the causes of gaps, customizing educational content, strengthening dermoscopy practices, providing psychological and communication skills, and providing continuous feedback and evaluation, we can effectively narrow the confidence gap between dermatologists when using dermoscopy, improve the level of dermatoscopic diagnosis and treatment, and increase patient satisfaction. This will help improve the service quality and patient safety level of the entire dermatology medical field.

We believe that the use of dermatoscopes should be promoted and popularized in western and remote areas of China in the future. By improving the education and professional certification of doctors, providing more opportunities for dermatoscopy training, simplifying access to dermatoscopy, and promoting dermatoscopy in grassroots hospitals, we can increase the confidence of dermatologists in the use of dermatoscopy in clinical diagnosis and treatment, thereby improving the diagnostic rate of skin diseases and improving the effectiveness of the treatment of skin diseases. From the perspective of future development trends, dermatoscopy will undoubtedly become a highly mature and promising auxiliary diagnostic method in the field of dermatology. In the future, more resources, including funding from national government departments, continuous attention from health authorities, the establishment of a team of skin imaging experts, and the gathering of resources from skin mirror‐related enterprises, are needed to further promote the application and rapid development of skin mirrors in the field of dermatology in China.

## Ethics Statement

This study was reviewed and approved by the Huashan Hospital Research Ethics Committee. The study protocol was approved by the Institutional Review Board of Huashan Hospital of Fudan University. This study is an online questionnaire survey. This study does not involve animal research or human research. This study does not belong to clinical trials.

The article "Multivariate Analysis and Prediction Model Construction for Dermatoscope Use by Chinese Dermatologists via an Online Survey" was published in 2024. Journal: Skin Res Technol.

## Consent for Publication

The authors provided consent for the publication of this article.

## Conflicts of Interest

There were no possible conflicts of interest.

## Data Availability

The data that support the findings of this study are available on request from the corresponding author. The data are not publicly available due to privacy or ethical restrictions.
